# The Effect of Humanized Nursing Intervention Guided by Computed Tomography Images on Elderly Patients Undergoing Anesthesia for Femur Intertrochanteric Fractures under Intelligent Reconstruction Algorithm

**DOI:** 10.1155/2022/5070518

**Published:** 2022-05-24

**Authors:** Yanfang He, Yufang Li, Rong Zeng, Xiaoyan Zhang

**Affiliations:** Department of Anesthesia Surgery Department, Changsha Fourth Hospital, Changsha, 410006 Hunan, China

## Abstract

This research was aimed at analyzing the effect of humanized nursing intervention combined with computed tomography (CT) imaging in the surgical anesthesia of femur intertrochanteric fractures (FIF) in the elderly. An image reconstruction algorithm was proposed based on nonlocal mean (NLM) algorithm, which was named as ONLM, and its performance was analyzed. A total of 114 elderly patients with FIF were equally and randomly divided into a humanized nursing group (57 cases) and a routine nursing group (57 cases). They were performed with CT imaging scan based on the ONLM algorithm, and the clinical indicators of the two groups of patients were recorded. The root mean square error (RMSE) and mean absolute error (MAE) of the CT images constructed using the ONLM algorithm were significantly lower than those using NLM algorithm, edge filtering algorithm, and total variation model, while the peak signal-to-noise ratio (PSNR) was the opposite (*P* < 0.05). The operation time, hospitalization days, intraoperative blood loss, postoperative drainage, and anesthesia preparation time of patients in the humanized nursing group were significantly lower than those in the routine nursing group. The number of patients with excellent Harris scores in the humanized nursing group was higher than that in the routine nursing group, and the number of patients with poor Harris scores was lower (*P* < 0.05). The language pain score, facial pain score, and visual analog simulation (VAS) scores of patients in the humanized nursing group were significantly lower than those in the routine nursing group. The numbers of postoperative hip varus and fracture nonunion cases in the humanized nursing group were significantly more than those in the routine nursing group. In short, CT images constructed by the ONLM showed higher performance than those by the traditional algorithm. In addition, CT images constructed by ONLM combined with humanized nursing intervention could more effectively improve the cooperation of patients with surgical anesthesia, reduce surgical pain and fear of patients, improve the prognosis of patients, and lower the occurrence of adverse events.

## 1. Introduction

Femur intertrochanteric fracture (FIF) refers to the fracture from the base of the femur neck to the level of the lesser trochanter, also known as intertrochanteric fracture, which accounts for 3% to 4% of all fracture types and 35.7% of hip fractures [1, 2]. FIF is generally more common in the elderly. The average age of patients is about 70 years old, which is about 6 years older than patients with femoral neck fractures. It is often caused by low-energy injuries. After FIF, it often causes hip pain, swelling, deformity, and limitation of movement [3–5]. If FIF is treated nonsurgically, it has many complications, and it is prone to complications such as pressure ulcers, lung infections, urinary tract infections, and deep vein thrombosis of the lower extremities, which can easily endanger the lives of patients [6]. Therefore, if the patient has no obvious surgical contraindications, for FIF, surgical treatment is recommended to stabilize the fracture end, shorten the patient's bedtime, and reduce the complications of the patient's bed [7, 8]. For patients undergoing surgical treatment, early rehabilitation training and functional exercise are required after surgery, which is beneficial to the rehabilitation of the function of the affected limb after fracture [9]. At present, the most commonly used surgical methods in clinical practice are locking plate internal fixation, dynamic hip screw(DHS) internal fixation, compression hollow nail internal fixation, and intramedullary nail internal fixation. Among them, intramedullary nail internal fixation is the most commonly used operation, which has the advantages of less trauma, reliable internal fixation, and low surgical failure rate [10].

Clinical imaging examination methods for FIF include plain X-ray film, CT, and magnetic resonance imaging (MRI). A plain radiograph can detect fractures. However, in some special fracture types (such as incomplete fractures and fatigue fractures), because the fracture has no displacement, there are only irregular fissures, which cannot be displayed on X-ray films. In addition, the major and minor trochanters of the femur, intertrochanteric line, crest, and soft tissue overlap on X-ray films, so fractures are easily missed [11]. MRI can clearly show incomplete fractures and fatigue fractures of femoral neck base or trochanter and intertrochanteric fissure fractures. It has obvious advantages, but its operation is more complicated and expensive [12]. CT can reduce the rate of missed diagnosis of femoral neck base or trochanter and intertrochanteric fissure fractures by X-ray, high-quality display of cortical bone continuity, and internal structure of bone slices, but there will be vascular shadow interference, missed scanning level, and other problems [13]. In order to improve the quality of the image, artificial intelligence technology is usually introduced to enhance the image processing [14]. The current reconstruction algorithms for CT images mainly include image domain reconstruction algorithms, projection data noise reduction algorithms, and postprocessing algorithms. Among them, the postprocessing algorithm does not need projection data, avoiding that the subsequent research cannot be carried out due to the lack of projection data. In addition, the storage space size and real-time requirements of the auxiliary system are lower, and it has a better development prospect [15].

In summary, the application of artificial intelligence algorithms and imaging technology in clinical surgical treatment is a promising direction. In this study, 114 elderly FIF patients were selected as the research objects. According to the different nursing plans, they were divided into a humanized nursing group and a routine nursing group. Only CT images based on artificial intelligence algorithms were used for inspection, and clinical indicators of patients were recorded, to explore the application value of humanized nursing intervention combined with CT images in anesthesia for elderly FIF surgery through comparative analysis, so as to provide a feasible solution for the clinical diagnosis and treatment of FIF.

## 2. Materials and Methods

### 2.1. Research Objects

A total of 114 elderly FIF patients who were treated in hospital from October 2016 to March 2021 were selected as the research subjects, including 43 males and 71 females. All patients underwent X-ray plain film, CT, hematuria, blood type, and blood cross test after admission. All subjects participated voluntarily and signed the informed consent forms, and this study was approved by the ethics committee of the hospital.

Inclusion criteria: patients >59 years old, patients with complete clinical data, patients who had not yet received treatment, and patients who voluntarily signed an informed consent form.

Exclusion criteria: patients with previous related department diseases, patients with surgical contraindications, patients with severe cardiopulmonary diseases, patients with coagulation disorders, and patients with poor blood sugar control.

### 2.2. Research Groups and Nursing Schemes

The patients were randomly divided into a humanized nursing group (57 cases) and a routine nursing group (57 cases).

Routine nursing group: the patients were conducted for health education before surgery, instruct patients to fast and water and other precautions, prepare for catheterization and skin test, etc.

Humanized nursing group: the patients were popularized for the relevant knowledge of surgical anesthesia, explain the entire procedure and safety of the operation, etc., to reduce the fear of the unknown of the patient facing the operation. Secondly, it had to pay attention to the patient's emotional changes in real time, actively communicate with the patient, relieve the patient's negative emotions, and improve treatment compliance. Thirdly, due to the pain and torture caused by the fracture to the patient, the nursing staff should help the patient carry out the traction of the affected limb to reduce the pain of the patient. During the operation, the patient should be presented in the most appropriate posture. Fourthly, during anesthesia, it could divert the patient's attention by chat and monitor the changes in the patient's vital characteristics. After the operation is completed, a soft pad was placed under the affected limb to reduce the pain caused by the shock or displacement involved in the wound when moving.

### 2.3. CT Examination

The CT scanning was performed with 64-slice spiral CT instrument. The patient was instructed to take a supine position, the lower limb of the unaffected side was in a straight state, and the patient was assisted in internal rotation of the affected limb by 15°. High-definition scanning was used to comprehensively scan the fracture site. The scanning range was from the anterior superior iliac spine to the middle of the femur, and the focus center was the proximal femur on the affected side. The scanning parameters were set as follows: the voltage was 130 kV, the current was 300 mA, the layer thickness was 0.521 mm, and the layer spacing was 0.521 mm.

### 2.4. Image Reconstruction Algorithm Based on Optimized Nonlocal Mean (ONLM)

The nonlocal mean (NLM) noise reduction algorithm was proposed by Buades et al. in 2005. This algorithm uses image block similarity and image redundancy for image denoising and reconstruction and has the advantages of strong detail retention and good filtering performance. It was supposed that a noise image was *P*, and then, below equation could be obtained:

(1) $$\begin{array}{c} P=\left\{P\left(i\right)\left|i\in \Theta \right.\right\},\\ P\left(i\right)=\underset{j\in U}{\sum }z\left(i,j\right)P\left(j\right). \end{array}$$

In the above two equations, Θ was the pixel set, *U* represented the search window, *P*_*i*_(*i*) represented the filtered pixel value at pixel *i*, *z*(*i*, *j*) represented the similarity between pixel *i* and pixel *j*, and 0 ≤ *z*(*i*, *j*) ≤ 1 and ∑_*j*_*z*(*i*, *j*) = 1. In order to further compare the similarity between pixel *i* and pixel *j*, the neighborhood was set as *M*, which was given as follows.

(2) $$\begin{array}{c} M={\left\{M_{i}\right\}}_{i\in I}, \end{array}$$

(3) $$\begin{array}{c} j\in M_{i}\Rightarrow i\in M_{j}. \end{array}$$

In equations (2) and (3), *M*_*i*_ was the similarity window, and the similarity window gray vector can be used to measure the similarity between pixel *i* and pixel *j*. Then, the Gaussian-weighted Euclidean distance was introduced to quantitatively calculate the similarity of the neighborhood corresponding to pixel *i* and pixel *j*, and below equation could be obtained:

(4) $$\begin{array}{c} l={\left\|P\left(M_{i}\right)-P\left(M_{j}\right)\right\|}_{2,\lambda }^{2}. \end{array}$$

In equation (4), *P*(*M*_*i*_) represented the area corresponding to pixel *i*, *P*(*M*_*j*_) represented the neighborhood corresponding to pixel *j*, *l* was the Gaussian-weighted Euclidean distance, and *λ* referred to the standard deviation of the Gaussian kernel, which was the weighted Gaussian kernel with *r* as the radius.

The calculation process of the Gaussian kernel [16] can be expressed as follows: it was supposed that the window radius was *r*, the variance was *λ*, and the window width was 2*r* + 1; then, below equation could be obtained:

(5) $$\begin{array}{c} K_{r}\left(i,j\right)=\exp\langle -\frac{{\left(j-r\right)}^{2}-{\left(i-r\right)}^{2}}{2\lambda^{2}}\rangle ,\\ \text{SUM}=K_{r}\left(i,j\right)+\text{SUM}. \end{array}$$

Loop calculations were performed until the end of the entire traversal. *K*_*r*_ in the above equations referred to the Gaussian kernel. Then, the Gaussian kernel was normalized as follows:

(6) $$\begin{array}{c} K_{r}=\frac{K_{r}}{\text{SUM}}. \end{array}$$

Then, the Gaussian Euclidean distance of the domains *P*(*M*_*i*_) and *P*(*M*_*j*_) can be expressed as follows:

(7) $$\begin{array}{c} L_{r}=K_{r}\overset{2r+1}{\underset{u=1}{\sum }}\overset{2r+1}{\underset{v=1}{\sum }}\left(P\left(M_{i}\right)\left(u,v\right)-P\left(M_{i}\right){\left(u,v\right)}^{2}\right),\\ L=L+L_{r}. \end{array}$$

In the above two equations, *L*_*r*_ represented the Gaussian Euclidean distance, and finally, the Euclidean-weighted distance of the pixel was calculated [17]:

(8) $$\begin{array}{c} l=\frac{L}{{\left(2r+1\right)}^{2}}. \end{array}$$

Then, the application of Euclidean-weighted distance in the field of noise can be expressed as

(9) $$\begin{array}{c} F{\left\|P\left(M_{i}\right)-P\left(M_{j}\right)\right\|}_{2,\lambda }^{2}={\left\|P*\left(M_{i}\right)-P*\left(M_{j}\right)\right\|}_{2,\lambda }^{2}+2\delta^{2}. \end{array}$$

In the above equation, *P*∗ represented the original image, and *δ*^2^ represented the noise variance. For most image blocks, the closer to the target pixel, the greater the weight, so the weight can be expressed as follows:

(10) $$\begin{array}{c} z\left(i,j\right)=\frac{\sum_{j}e^{\left(-{\left\|P\left(M_{i}\right)-P\left(M_{j}\right)\right\|}_{2,\lambda }^{2}/\kappa^{2}\right)}}{\beta \left(i\right)}, \end{array}$$

(11) $$\begin{array}{c} \beta \left(i\right)=\underset{j\in M}{\sum }\exp\langle -\frac{{\left\|P\left(M_{i}\right)-P\left(M_{j}\right)\right\|}_{2,\lambda }^{2}}{\kappa^{2}}\rangle . \end{array}$$

In equations (10) and (11), *β*(*i*) represented the normalization factor, and *κ* determined the parameter of the degree of filtering. However, the above algorithm tended to ignore the difference between the gray values of pixel neighborhoods when the weights were calculated, resulting in blurred edges. When *z*(*i*, *j*) = max*z*(*i*, *j*) and *i* ≠ *j*, the Gaussian preprocessing was performed on the image [18]. A template size was set to (2*h* + 1)∗(2*h* + 1), and then, the element size in the Gaussian template can be calculated with below equation:

(12) $$\begin{array}{c} K_{\delta }\left(x,y\right)=\frac{\exp\langle -\left(\left(x^{2}+y^{2}\right)/2\delta^{2}\right)\rangle }{2{\pi \delta }^{2}}. \end{array}$$

In the equation above, (*x*, *y*) = {−*h*, ⋯, h}, and *δ* represented Gaussian standard deviation. Then, the below equations could be obtained after the normalization process:

(13) $$\begin{array}{c} \text{SUMK}=\overset{h}{\underset{x=-h}{\sum }}\overset{h}{\underset{y=-h}{\sum }}K_{\delta }\left(x,y\right), \end{array}$$

(14) $$\begin{array}{c} {DK}_{\delta }\left(x,y\right)=\frac{K_{\delta }\left(x,y\right)}{\text{SUMK}}. \end{array}$$

In equation (14), *DK*_*δ*_ represented the Gaussian filter. Then, for each image block, after Gaussian filtering, below equation could be acquired:

(15) $$\begin{array}{c} P_{K}\left(M_{i}\right)={DK}_{\delta }\left(i\right)\cdot P\left(M_{i}\right). \end{array}$$

In equation (15), *P*_*K*_(*M*_*i*_) represented the result of each image block processed by Gaussian filtering. It was assumed that the horizontal gradient and vertical gradient of the central pixel of the image were $\bar{s_{x}}$ and $\bar{s_{y}}$, respectively, which can be expressed as below equations:

(16) $$\begin{array}{c} \bar{s_{x}}=\frac{\left|s\left(x,y\right)-s\left(x,y-1\right)\right|+\left|s\left(x,y\right)-s\left(x,y+1\right)\right|}{2},\\ \bar{s_{y}}=\frac{\left|s\left(x,y\right)-s\left(x-1,y\right)\right|-\left|s\left(x,y\right)-s\left(x+1,y\right)\right|}{2}. \end{array}$$

Similarly, the average gradient of the neighborhood of pixel *i* can be given as follows:

(17) $$\begin{array}{c} \bar{\Delta s}\left(i\right)=\langle \bar{s_{x}}\left(i\right),\bar{s_{y}}\left(i\right)\rangle . \end{array}$$

Then, the angle Angle(*i*, *j*) between the average gradient of the neighborhood of pixels *i* and *j* could be calculated:

(18) $$\begin{array}{c} \text{Angle}\left(i,j\right)=∡\langle \bar{s}\left(i\right),\bar{s}\left(j\right)\rangle . \end{array}$$

Then, the weight of the improved algorithm can be expressed as follows:

(19) $$\begin{array}{c} P\left(i\right)=\underset{j\in M}{\sum }Z_{K}\left(i,j\right)P_{K}\left(j\right),\\ Z_{K}\left(i,j\right)=\frac{e^{\left(-{\left\|P_{K}\left(M_{i}\right)-P_{K}\left(M_{j}\right)\right\|}_{2,\lambda }^{2}/{\kappa_{1}}^{2}\right)-\left({\left\|M_{i}-M_{j}\right\|}_{2,\lambda }^{2}/{\kappa_{2}}^{2}\right)-\left(\text{Angle}\left(i,j\right)/\tau^{2}\right)}}{\beta \left(i\right)},\\ \beta \left(i\right)=\underset{j\in M}{\sum }\exp\langle -\frac{{\left\|P_{K}\left(M_{i}\right)-P_{K}\left(M_{j}\right)\right\|}_{2,\lambda }^{2}}{{\kappa_{1}}^{2}}-\frac{{\left\|M_{i}-M_{j}\right\|}_{2,\lambda }^{2}}{{\kappa_{2}}^{2}}-\frac{\text{Angle}\left(i,j\right)}{\tau^{2}}\rangle ,\\ {\kappa_{1}}^{2}=\alpha *\text{mean}{\left\|P_{K}\left(M_{i}\right)-P_{K}\left(M_{j}\right)\right\|}_{2,\lambda }+c. \end{array}$$

In the above equations, *P*_*K*_(*j*) represented the Gaussian filtered image, *Z*_*K*_ represented the optimized weight function, ‖*P*_*K*_(*M*_*i*_) − *P*_*K*_(*M*_*j*_)‖_2,*λ*_^2^/*κ*_1_^2^ represented the spatial proximity factor, ‖*M*_*i*_ − *M*_*j*_‖_2,*λ*_^2^/*κ*_2_^2^ referred to the gray-scale similarity factor, Angle(*i*, *j*)/*τ*^2^ represented the adjustment function of the neighborhood gradient direction difference, *τ* was the filter parameter, *κ*_1_ was the spatial distance adjustment parameter, *κ*_2_ was the grayscale spatial distance adjustment parameter, *α* was the filter degree adjustment parameter, and *c* referred to the balance parameter of the image noise reduction strength. In this study, the optimized NLM noise reduction algorithm was recorded as ONLM.

### 2.5. Objective Evaluation Indicators

The root mean square error (RMSE), mean absolute error (MAE), and peak signal-to-noise ratio (PSNR) were used to evaluate the effect of the algorithm on image reconstruction.

The size of an image was supposed as *Q*_1_ × *Q*_2_, and then, below equations could be obtained:

(20) $$\begin{array}{c} \text{RMSE}=\sqrt{\frac{\sum_{i=1}^{Q_{1}}\sum_{j=1}^{Q_{2}}{\left|H_{0}\left(i,j\right)-H_{1}\left(i,j\right)\right|}^{2}}{Q_{1}*Q_{2}}},\\ \text{MAE}=\frac{\sum_{i=1}^{Q_{1}}\sum_{j=1}^{Q_{2}}\left|H_{0}\left(i,j\right)-H_{1}\left(i,j\right)\right|}{Q_{1}*Q_{2}},\\ \text{MSE}=\frac{\sum_{i=1}^{Q_{1}}\sum_{j=1}^{Q_{2}}{\left|H_{0}\left(i,j\right)-H_{1}\left(i,j\right)\right|}^{2}}{Q_{1}*Q_{2}},\\ \text{PSNR}=10\mathrm{lg}\frac{255*255}{\text{MSE}}. \end{array}$$

In the above equations, *H*_0_(*i*, *j*) was the pixel value of the original image in (*i*, *j*), and *H*_1_(*i*, *j*) was the pixel value of the reconstructed image.

The traditional NLM algorithm, the bilateral filter algorithm [19], and the total variation (TV) model [20] were introduced to compare with the ONLM algorithm in this study.

### 2.6. Observation Indicators

The age, male/female ratio, body mass index (BMI), Evans-Jensen classification, and type of surgery (dynamic hip screw, proximal femoral antirotation intramedullary nail, and Medoff sliding compression plate) were recorded for the two groups of patients. The surgical indicators (operation time, hospitalization time, intraoperative blood loss, postoperative drainage, and anesthesia preparation time) of the two groups of patients were recorded. The visual analogue scale (VAS), language pain score, and facial expression pain score were used to assess the degree of pain before and after nursing. It should follow up and record the adverse events of the two groups of patients after the operation.

### 2.7. Statistical Methods

The data in this study was analyzed by SPSS19.0 version statistical software, the measurement data was expressed as the mean ± standard deviation ($\overset{¯}{x}\pm s$), and the count data was expressed as the percentage (%). Pairwise comparison adopted one-way analysis of variance. The difference was statistically significant at *P* < 0.05.

## 3. Results

### 3.1. Image Reconstruction Results Using Four Algorithms

Figure 1 shows the image reconstruction results of the four algorithms. The four algorithms had significantly improved the quality of CT images. Among them, the NLM algorithm, edge filtering algorithm, and TV model effectively remove the noise of the original image, but there were still some streak artifacts. The ONLM algorithm reconstructed the image most clearly, the noise and artifacts were greatly reduced, and the image details were kept intact.

In terms of objective evaluation (Figure 2), the RMSE and MAE levels of the reconstructed image of the ONLM algorithm were significantly lower than those of the NLM algorithm, edge filtering algorithm, and total variation model, and the differences were statistically significant (*P* < 0.05). The PSNR level of the reconstructed image of ONLM algorithm was significantly higher than that of NLM algorithm, edge filtering algorithm, and total variation model, and the difference was statistically significant (*P* < 0.05).

### 3.2. Comparison of Basic Information of the Two Groups of Patients

As shown in Figure 3, the age, male/female ratio, BMI, Evans-Jensen classification, age, type of operation (dynamic hip screw, proximal femoral antirotation intramedullary nail, and Medoff sliding compression plate), and time from injury to operation of patients in the humanized nursing group and routine nursing group showed no obvious difference (*P* > 0.05).

A 60-year-old male patient was admitted to the hospital with the chief complaint of “pain in the left hip for 3 days after a fall”, as shown in Figure 4. CT examination showed that the left hip fracture was sclerotic, the adjacent soft tissue layers were unclear, and there were signs of swelling. A left hip fracture was diagnosed.

### 3.3. Comparison of Surgical Indicators between the Two Groups

As shown in Figure 5, the operation time, hospitalization time, intraoperative blood loss, postoperative drainage, and anesthesia preparation time of the humanized nursing intervention group were significantly lower than those of the routine nursing group, and the differences were statistically significant (*P* < 0.05).

### 3.4. Comparison of Postoperative Hip Scores between the Two Groups

As shown in Figure 6, the number of patients with excellent Harris scores in the humanized nursing intervention group was significantly higher than that in the routine nursing group, and the difference was statistically significant (*P* < 0.05). The number of patients with poor Harris scores in the humanized nursing intervention group was obviously lower than that in the routine nursing group, showing statistically significant difference (*P* < 0.05).

### 3.5. Comparison of Pain Scores between the Two Groups of Patients before and after Nursing

As shown in Figure 7, the differences in language pain score, facial pain score, and VAS scores of the two groups before nursing were not statistically significant (*P* > 0.05). The language pain score, facial pain score, and VAS scores of the humanized nursing group after nursing were significantly lower than those of the routine nursing group, and the differences were statistically significant (*P* < 0.05).

### 3.6. Comparison of Adverse Events between the Two Groups of Patients

As shown in Figure 8, in the humanized nursing group, there were 2 cases of deep venous thrombosis in the lower limbs, 1 case of hip varus, 1 case of fracture nonunion, and 2 cases of ipsilateral thigh pain. In the routine nursing group, there were 2 patients of deep venous thrombosis of the lower extremities, 3 patients of hip varus, 4 patients of fracture nonunion, and 2 patients of affected thigh pain. Among them, the number of hip varus and fracture nonunion patients in the humanized nursing group was significantly more than that in the routine nursing group, and the difference was statistically significant (*P* < 0.05). Compared with routine nursing group, the number of patients with deep vein thrombosis of lower extremity and the number of patients with pain in the ipsilateral thigh after operation was not statistically significant (*P* > 0.05).

## 4. Discussion

As the largest bone of the human body, the femur is an important part to support the normal movement of the body. The occurrence of FIF will not only affect the basic mobility of the patient but also lose the ability to take care of itself. Long-term bed rest can also lead to a series of complications. Therefore, targeted care is needed during surgical treatment to improve the patient's recovery and prognosis [21, 22]. In order to improve the image quality, an image reconstruction algorithm (ONLM) based on optimized NLM was proposed and compared with several traditional algorithms in this work. It can be found that the ONLM algorithm reconstructed the image most clearly, the noise and artifacts were greatly reduced, the image details were kept intact, and the overall quality was better than the NLM algorithm, edge filtering algorithm, and total variation model. After further comparison of the objective evaluation indicators of the algorithm, it was found that the RMSE and MAE levels of the reconstructed image of the ONLM algorithm were significantly lower than those of the NLM algorithm, edge filtering algorithm, and total variation model, while the PSNR level was significantly higher than NLM algorithm, edge filtering algorithm, and total variation model (*P* < 0.05). Such results are similar to the research on artificial intelligence algorithms by Chen and Kim [23], which shows that the ONLM algorithm has excellent performance in denoising and reconstruction of CT images and is worthy of popularization and application.

The optimized algorithm was applied to clinical research. In this study, 114 elderly FIF patients were divided into a humanized nursing group (57 cases) and a routine nursing group (57 cases), and the clinical indicators of the two groups of patients were recorded. Firstly, it was found that the operation time, hospitalization time, intraoperative blood loss, postoperative drainage, and anesthesia preparation time of the humanized nursing intervention group were significantly lower than those of the routine nursing group, and the differences were statistically significant (*P* < 0.05). This shows that compared with routine nursing, humanized nursing intervention can effectively improve the cooperation of patients with surgical anesthesia, thereby shortening the postoperative hospitalization time of patients and speeding up the recovery of patients [24]. The number of patients with excellent Harris score in the humanized nursing intervention group was higher than that in the routine nursing group, and the number of patients with poor Harris score was lower than that of the routine nursing group (*P* < 0.05). Harris score is a widely used method to evaluate hip joint function. It is often used to evaluate the effect of postoperative hip preservation. The results show that humanized nursing can effectively improve the recovery of the hip joint after surgery [25]. The language pain score, facial pain score, and VAS scores of the humanized nursing group after nursing were significantly lower than those of the routine nursing group, and the difference was statistically significant (*P* < 0.05). Surgical analgesia for patients has always been a problem that needs clinical attention. Humanized nursing takes the patient as the core and can intervene in many aspects such as patient cognition and psychology [26]. This shows that humanized nursing can reduce the patient's surgical pain to a certain extent and ensure the orderly progress of surgical treatment. The number of hip varus and fracture nonunion patients in the humanized nursing group was significantly more than that in the routine nursing group, and the difference was statistically significant (*P* < 0.05). It shows that humanized nursing intervention can effectively improve the prognosis of patients and reduce the occurrence of adverse events. Most of the previous studies focused on single algorithm and imaging or the effects of emerging nursing methods in clinical practice. The innovation of this work was to combine the CT examination based on the ONLM algorithm with humanized nursing intervention, which was applied to patients with FIF, aiming to provide a sustainable reference basis and future research ideas for the clinical diagnosis and treatment of the FIF.

## 5. Conclusion

In this research, the ONLM, an image reconstruction algorithm based on optimized NLM algorithm, was applied in CT examinations of elderly patients with FIF. The results showed that, compared with routine nursing, CT image-based guidance with humanized nursing intervention can more effectively improve the cooperation of patients with surgical anesthesia, reduce surgical pain and fear of patients, improve the prognosis of patients, and lower the occurrence of adverse events. However, it did not separately compare patients of different types of surgery, which may affect the results slightly. In addition, the follow-up time was relatively short, and a more detailed group study would be considered later. In short, the results of this work provided a data reference for the feasibility of clinical surgical treatment combined with nursing intervention for surgical anesthesia for patients with FIF.

## Figures and Tables

**Figure 1:** Image reconstruction results of four algorithms. (a) was the original image; (b)–(e) showed the images reconstructed by NLM algorithm, edge filtering algorithm, total variation model, and ONLM algorithm, respectively.

**Figure 2:** Comparison of the objective evaluation indicators of the four algorithms to reconstruct the image. (a), (b), and (c) showed the comparisons of MAE, PSNR, and RMSE, respectively. ∗ indicated that the difference compared with ONLM algorithm was statistically significant (*P* < 0.05).

**Figure 3:** Comparison of basic data of subjects in the humanized nursing group and routine nursing group. (a) showed the comparison of age, male/female ratio, and BMI; (b) showed the comparison on Evans-Jensen classification; (c) showed the comparison on the type of surgery (dynamic hip screw, proximal femoral antirotation intramedullary nail, and Medoff sliding compression plate); and (d) showed the comparison on time from injury to operation.

**Figure 4:** CT image of the left hip of a 60-year-old man.

**Figure 5:** Comparison of surgical indicators between the two groups. (a) showed the comparison of operation time and hospitalization time; (b) showed the comparison of intraoperative blood loss and postoperative drainage; and (c) showed the comparison of anesthesia preparation time. ∗ indicated that the difference was statistically significant compared with the humanized nursing group (*P* < 0.05).

**Figure 6:** Comparison of postoperative hip scores between the two groups. ∗ indicated that the difference was statistically significant compared with the humanized nursing group (*P* < 0.05).

**Figure 7:** Comparison of pain scores between the two groups of patients before and after nursing. (a) showed the comparison of language pain score; (b) showed the comparison of facial pain score; and (c) showed the comparison of VAS score. ∗ indicated that the difference was statistically significant compared with the humanized nursing group (*P* < 0.05).

**Figure 8:** Comparison of adverse events between the two groups of patients. ∗ indicated that the difference was statistically significant compared with the high-intensity group (*P* < 0.05).

## Data Availability

The data used to support the findings of this study are available from the corresponding author upon request.
